The article "Implementation of Postpartum Hemorrhage Emergency Care Using a Bundle Approach at a Tertiary Care Hospital in North India" was retracted in 2022. Reasons: errors in the text; concerns about the authorship.

# Implementation of Postpartum Hemorrhage Emergency Care Using a Bundle Approach at a Tertiary Care Hospital in North India

**DOI:** 10.7759/cureus.26819

**Published:** 2022-07-13

**Authors:** Singh Jigyasa, Sakshi Agrawal, Uma Pandey, Shikha Sachan, Mamta Rajan, Tej Bali Singh, Surabhi Sapna

**Affiliations:** 1 Obstetrics and Gynecology, Institute of Medical Sciences Banaras Hindu University (IMS BHU), Varanasi, IND; 2 Preventive Medicine, Institute of Medical Sciences Banaras Hindu University (IMS BHU), Varanasi, IND

**Keywords:** postpartum hemorrhage, blood transfusion, maternal morbidity, implementation, care bundle, postpartum haemorrhage

## Abstract

Background

The major cause of maternal death globally is postpartum hemorrhage (PPH). When PPH develops, early detection of bleeding and rapid treatment with evidence-based guidelines can prevent most PPH-related severe morbidity and mortality. The bundle care approach for PPH management could be a potential solution to inefficient and uneven evidence-based practice implementation worldwide. Bundle care is a collection of discrete, evidence-based interventions given to every eligible person simultaneously or in quick succession and requires teamwork, communication, and cooperation. The primary objective of this study was to analyze whether implementing a PPH bundle of care may reduce maternal morbidity and mortality in our institution.

Methods

This was a single-center retrospective pre-post case-control study was carried out at a tertiary care center and teaching hospital in Varanasi, eastern Uttar Pradesh state, India. From January 2021 to June 2021, pretraining data (PRE) were collected retrospectively on all births from the department of Obstetrics and Gynecology, Sir Sunderlal Hospital, Institute of Medical Sciences, Banaras Hindu University. Subsequently, medical and paramedical personnel of our hospital were trained in Postpartum Hemorrhage Emergency Care Using a Bundle Approach (PPH EmC) as per the guidelines laid down by the World Health Organization (WHO) for PPH management and implemented in July 2021. Post-training data (POST) were then collected retrospectively on all deliveries at our hospital from August 2021 to January 2022. All the data within two periods were computed and analyzed. The results were then compared for any significant changes in the incidences of maternal mortality and morbidity in terms of the rates of blood transfusion required and the type of management used (medical or medical-surgical), use of tranexamic acid, and additional uterotonics. The results were expressed as proportions, and p≤0.05 was considered statistically significant using IBM SPSS Statistics for Windows, version 24.0 (IBM Corp., Armonk, NY, USA).

The article "Implementation of Postpartum Hemorrhage Emergency Care Using a Bundle Approach at a Tertiary Care Hospital in North India" was retracted in 2022. Reasons: errors in the text; concerns about the authorship.

Results

A total of 1304 women gave birth from January 2021 to January 2022, of whom 107 patients (61 in the PRE and 57 in the POST group) were diagnosed and treated for PPH. There was no significant difference in the incidence of PPH in the PRE and POST groups (p=0.581). There was a significant increase in the use of tranexamic acid (p=0.041) and a significant reduction in blood transfusion rates (p=0.032) after the implementation of bundled care in the POST group. The odds of PPH non-occurrence after pre- and post-test was 1.103 (95% CI=0.747 to 1.635). No significant difference was observed in maternal mortality in the PRE and POST groups (p=0.96). The requirement for radical surgical treatment of PPH, which included hysterectomies, was also significantly reduced, from 27.27% in the PRE group to 11.54% in the POST group (p=0.032).

Conclusions

PPH care bundles might improve the morbidity of PPH with the use of fewer resources and fewer interventions required. While these data are promising, further studies are needed to analyze bundle care's long-term effects.

## Introduction

With an estimated mortality rate of 140,000 per year (i.e., one maternal death every four minutes), postpartum hemorrhage (PPH) remains a significant cause of maternal mortality and morbidity worldwide, particularly in low-income countries [1]. PPH occurs in 5% of all deliveries, and most deaths occur within four hours of delivery, indicating that PPH is a consequence of the third stage of labor [2].

Worldwide, approximately half a million women die due to complications of pregnancy and childbirth. Nearly all of these deaths (99%) occur in low and middle-income nations. Despite having only 16% of the world's population, India accounts for almost 20% of maternal mortality. PPH is a common delivery complication, with rates ranging from 2% to 6% after vaginal delivery and 6% after cesarean section, with uterine atony accounting for roughly half of the cases. In poorer nations, it accounts for 28% of all maternal deaths [2].

Numerous factors contribute to PPH, including uterine atony, a prolonged third stage of labor, a retained placenta, pregnancy-induced hypertension, anemia, and history of PPH, uterine rupture, abruptio placenta, placenta previa, and maternal coagulation abnormalities [3,4]. Moreover, other factors include the number of pregnancies, number of fetuses, mode of delivery, lack of antenatal care, not receiving adequate nutritional supplementation, and any tear or injury to the genital tract [5-7].

PPH, which is aggravated by prevalent anemia among pregnant women in India, accounts for 38% of maternal mortality, according to the Sample Registration System report by the Registrar General of India [8]. The loss of a smaller blood volume may still result in adverse clinical sequelae. PPH describes a blood loss of 500 mL or more within 24 hours of giving birth or a minor blood loss that causes the woman to become hemodynamically unstable.

The article "Implementation of Postpartum Hemorrhage Emergency Care Using a Bundle Approach at a Tertiary Care Hospital in North India" was retracted in 2022. Reasons: errors in the text; concerns about the authorship.

According to the 2017 World Health Organization (WHO) guidance, treatment of PPH due to uterine atony consists of two major elements: first-response bundles, such as uterotonic drugs (mainly oxytocin), isotonic crystalloids, tranexamic acid (TXA), and uterine massage; and, if necessary, response to refractory PPH bundles, such as compressive measures (aortic compression or bimanual uterine compression), intrauterine balloon tamponade, and non-pneumatic anti-shock garment [9]. If these procedures are ineffectual, surgical intervention (such as compressive sutures, artery ligation, or hysterectomy) is required [10].

To improve the management of PPH patients, community and health care workers should be appropriately trained and counseled on the danger signs of pregnancy and early detection of high-risk pregnancies, timely diagnosis, and accurate estimation of blood loss following childbirth. However, the Federation of Obstetric and Gynecological Societies of India and other experts suggest a few additional key considerations for preventing and managing PPH at the community and facility level. In recent years, treatment bundles have been used to give high-quality clinical care by driving compliance with selected best practices and procedural improvements. The Massachusetts General Hospital Global Health Innovation Lab (MGH GHI) has partnered with leading obstetricians and maternal health champions worldwide to develop a comprehensive initiative to give high-quality PPH emergency care using a bundle strategy. PPH Emergency Care Using a Bundle Approach (EmC) incorporates critical clinical and systems-based treatments for prompt, efficient care [9,11].

There is little evidence regarding the challenges in the implementation of care bundle in low- and middle-income countries, particularly in maternal health and emergency settings, including factors like a lack of qualified staff, lack of essential supplies or medications, and overburdened services. Therefore, we conducted this study to analyze whether implementing a PPH bundle of care may reduce maternal morbidity and mortality in our institution.

## Materials and methods

Study design and setting

This retrospective, pre-post, case-control study was conducted at a tertiary care center and teaching hospital under the Banaras Hindu University in the eastern zone of the state of Uttar Pradesh, India.

The article "Implementation of Postpartum Hemorrhage Emergency Care Using a Bundle Approach at a Tertiary Care Hospital in North India" was retracted in 2022. Reasons: errors in the text; concerns about the authorship.

Ethical clearance and informed consent

The study design and protocol were approved by the Institutional Ethical Committee at the Institute of Medical Sciences, Banaras Hindu University (Reference Number EC/3225). Informed written consent was obtained from all the patients and family members to participate in the study.

Study duration

This study spanned a total duration of 13 months, starting from January 1, 2021, to January 31, 2022.

Study participants

*Inclusion Criteria* All women who developed PPH within the first 24 hours of delivery were included in the study.

*Exclusion Criteria* Women who developed late or secondary PPH and those who presented with first-trimester bleeding were not included in the study. Patients not willing to participate were excluded from the study as well.

Study size

Non-probability convenience sampling technique was used to enroll subjects in the study after careful assessment of the inclusion and exclusion criteria to arrive at the final sample size.

Independent variables

These included the demographic parameters, namely, gestational age, parity, gestation, associated diagnosis (cause of PPH), whether the patient was admitted or a referred case, the severity of the PPH developed, the mode of delivery (spontaneous vaginal delivery or cesarean), and the order of cesarean delivery (primary or repeat).

Outcome variables

The outcomes were assessed in terms of the dependent variables, which were as follows: shock index at the time of admission, the type of management required, the use of additional uterotonics and tranexamic acid, the need for blood transfusions and blood components, and the need for radical operations.

Data collection and follow-up

We compared the mortality and morbidity of PPH patients six months prior to Postpartum Hemorrhage Emergency Care Using a Bundle Approach (PPH EmC) training conducted in July 2022. That is, pre-training data (PRE) was collected via a retrospective review of delivery records from January 2021 to June 2021 from the institutional database. Subsequently, the post-training data (POST) was obtained for the deliveries in the six months following the training, that is, from August 2021 to January 2022.

We documented any volume of blood loss following birth that adversely influenced the mother, that is, losses of >500 mL in vaginal deliveries, and losses of >1000 mL in cesarean sections. Blood loss was measured objectively and subjectively in the hospital (calculated based on the use of sponges and the blood suctioned by the attending personnel). Mild PPH was defined as blood loss of 500 mL to 700 mL, moderate as 700 mL to 1000 mL, and severe PPH as any loss >1000 mL of blood. The criteria for diagnosing deliveries outside the institute were unclear, but as they were referred with a diagnosis of PPH from their primary treatment center and most of them were in a moribund state, no detailed description was sought for such delivery cases. These women were identified, and all case files were reviewed with demographic information such as age, parity, gestational period, and mode of birth. Shock index (SI), calculated as the heart rate divided by systolic blood pressure, was documented for all patients at admission and at regular time intervals according to the defined protocols at our institution. SI is a marker of hemodynamic status in patients with hypovolemic shock who need transfusions or massive transfusions as a marker of morbidity. An acceptable SI ranges from 0.5 to 0.9, while values approaching 1.0 are indicative of worsening hemodynamic conditions and shock requiring activation of the transfusion protocol [12]. The cause of the PPH and the medical or surgical interventions provided, the associated maternal morbidities, and related mortalities were analyzed. Since the data were collected retrospectively from the institutional registries after the fact, there wasn't much that could be done to amend bias.

The article "Implementation of Postpartum Hemorrhage Emergency Care Using a Bundle Approach at a Tertiary Care Hospital in North India" was retracted in 2022. Reasons: errors in the text; concerns about the authorship.

The PPH EmC was rolled out in several phases of training. In the first phase, the International Federation of Gynecology and Obstetrics of London, the Massachusetts General Hospital Global Health Innovation (MGH GHI) of the USA, and the Uttar Pradesh Technical Support Unit, in coordination with the Mahatma Gandhi Institute of Medical Sciences (MG IMS) in India, conducted training of trainer (TOT) sessions under the Bill and Melinda Gates Foundation-funded project "Engaging National Professional Societies to Combat Postpartum Hemorrhage," which aims to reduce maternal morbidity and mortality through the implementation of the PPH EmC program. In the second phase, staff nurses, resident doctors, obstetrics scrub nurses, and the labor room nursing assistants of our hospital were trained. In the third phase, which happened in December 2021, nurses and doctors from district hospitals, community health centers, and primary health centers other than our hospital were trained.

All the women were followed up for a minimum period of two months.

Statistical analysis

We produced descriptive statistics for the variables to define the population's demographic profile. Tests of normalcy were used to determine the normality of the data distribution. The categorical variables are expressed as proportions, and the groups were compared using the Chi-square test or Fisher's exact probability test. We considered p≤0.05 as significant. We used IBM SPSS Statistics for Windows, Version 24.0 (IBM Corp., Armonk, NY, USA) to analyze the data.

The article "Implementation of Postpartum Hemorrhage Emergency Care Using a Bundle Approach at a Tertiary Care Hospital in North India" was retracted in 2022. Reasons: errors in the text; concerns about the authorship.

## Results

A total of 1304 women gave birth between January 2021 and January 2022 (641 births in the PRE and 663 births in the POST time era), of whom 118 were diagnosed with PPH (frequency of PPH=9.1%). Sixty-one patients with PPH were admitted during the PRE period and 57 during the POST period. The incidence of PPH in the PRE group was 9.5% (95% CI=7.5% to 12.0%) and in the POST group was 8.6% (95% CI=6.6% to 11.0%). No significant difference was observed between the two groups (χ^2^=0.22, p=0.581). Complete data was not available for six patients in the PRE group and five patients in the POST group. Therefore, for further analysis, the PRE group consisted of 55 patients, and the POST group consisted of 52 patients.

The sociodemographic properties of the patients are summarized in Table 1.

**Table 1:** Demographic variables of patients with PPH Abbreviations: PPH, postpartum hemorrhage; PROM, premature rupture of membrane; PRE, pretraining data; POST, post-training data; G2, gravida 2; G3, gravida 3; G4, gravida 4.

Variable		PRE (n=55), n (%)	POST (n=52), n (%)	p-Value
Gestational age	<28 weeks	3 (5.45%)	3(5.77%)	0.995
	28–32 weeks	6 (10.91%)	5 (9.62%)	
	32–36 weeks	11 (20%)	10 (19.23%)	
	>36 weeks	35 (63.63%)	34 (65.38%)	
Parity	Primigravida	23 (41.81 %)	27 (51.92%)	0.356
	G 2	12 (21.81%)	11 (21.15%)	
	G 3	18 (32.72%)	10 (19.23%)	
	G 4	2 (3.63 %%)	4 (7.69%)	
Gestation	Singleton	54 (98.18%)	51 (98.08%)	1
	Twins	1 (1.82%)	1 (1.92%)	
Diagnosis	Severe anaemia	22 (40%)	18 (34.62%)	0.99
	Hypertensive disorders of pregnancy	8 (14.55%)	7 (13.46%)	
	Maternal sepsis	5 (9.09%)	4 (7.69%)	
	PROM	6 (10.90%)	7 (13.46%)	
	Thrombocytopenia	5 (9.09%)	6 (11.54%)	
	Antepartum hemorrhage	4 (7.27%)	5 (9.09%)	
	Preterm labor	3 (5.45%)	3 (5.77%)	
	Other	2 (3.6%)	2 (3.85%)	
Distribution of Admitted/Referral patients	Admitted patient	40 (72.72%)	41 (78.84%)	0.46
	Referred patient	15 (27.27%)	11 (21.15%)	
Severity of PPH	Mild	29 (52.72%)	32 (61.53%)	0.021
	Moderate	10 (18.18%)	1 (1.92%)	
	Severe	16 (29.09%)	19 (36.54%)	

Thirty-five PRE patients (63.6%) and 34 POST patients (65.4%) were admitted with a gestational age of >36 weeks. Twenty-three PRE patients (41.8%) and 27 POST patients (51.9%) were primigravida (χ2=3.23; p=0.35). Most of the patients from both periods had singleton pregnancies. Severe anemia was the most common condition in both periods, followed by pregnancy-induced hypertension and premature rupture of membrane. Mild PPH was most common in the PRE group (n=29, 52.7%), while 10 patients (18.2%) had moderate PPH, and 16 patients (29%) had severe PPH. In the POST group, mild PPH was the most common (n=32, 61.5%) followed by severe PPH (n=19, 36.5%); one patient in the POST group had moderate PPH (χ2=7.69; p=0.021). In the PRE group, 27 patients (49.1%) were aged 20 to 25 years, 23 (41.8%) were aged 26 to 30 years, and five (9.1%) were aged 31 to 35 years. In the POST group, 25 patients (48.1%) were aged 20 to 25 years, 21 (40.4%) were aged 26 to 30 years, and six (11.5%) were aged 31 to 35 years. Fifteen PRE patients (27.3%) and 11 POST patients (21.15%) were referred to our institution from a primary health center, community health center, district hospitals, or private hospitals. The maximum number of PPH patients from both groups (72.7% in the PRE group and 78.8% in the POST group) were booked in our hospital outpatient department or admitted directly to the emergency labor room.

The article "Implementation of Postpartum Hemorrhage Emergency Care Using a Bundle Approach at a Tertiary Care Hospital in North India" was retracted in 2022. Reasons: errors in the text; concerns about the authorship.

The mode of delivery is presented in Table 2.

**Table 2:** Delivery of patients with PPH Abbreviations: PPH, postpartum hemorrhage; SVD, spontaneous vaginal delivery; CD, cesarean delivery; PRE, pretraining data; POST, post-training data.

		PRE (n=55), n (%)	POST (n=52), n (%)	p-Value
Mode of delivery	SVD	32 (58.2%)	28 (53.8%)	0.65
	CD	23 (41.8%)	24 (46.1%)	
Order of Cesarean delivery	Primary	15 (65.2%)	14 (58.3%)	0.63
	Repeat	8 (34.8%)	10 (41.7%)	

Spontaneous delivery was most common in both PRE (n=32, 58.2%) and POST (n=28, 53.8%) groups. Twenty-three patients (41.8%) in the PRE group and 24 patients (46.1%) in the POST group required cesarean section. Primary cesarean delivery was common in both groups (χ2=0.235; p=0.63).

Table 3 presents an analysis of the interventions to manage PPH.

**Table 3:** Interventions done in the management of PPH Abbreviations: PPH, postpartum hemorrhage; PRBC, packed red blood cells; FFP, fresh frozen plasma; PRE, pretraining data; POST, post-training data.

		PRE (n=55), n (%)	POST (n=52), n (%)	p-Value
PPH etiology	Atonicity	50 (90.91%)	43 (82.69%)	0.47
	Trauma	3 (5.45%)	4 (7.69%)	
	Tissue	1(1.82%)	4 (7.69%)	
	Coagulation disorders	1 (1.82%)	1 (1.92%)	
Management	Medical alone	28 (50.91%)	34 (68.38%)	0.186
	Medical and surgical both	27 (49.09%)	18 (34.62%)	
Use of additional uterotonics		5 (9.1%)	5 (9.6%)	1
Use of tranexamic acid		7 (12.72%)	17 (32.69%)	0.041
Blood transfusion and components	PRBC	22 (40%)	15 (28.85%)	0.032
	FFP	5 (9.09%)	1 (1.92%)	
	PRBC + FFP	27 (49.09%)	4 (7.69%)	
Blood transfusion >4 units of PRBC		3 (5.45%)	4 (7.69%)	0.71
Radical operation (hysterectomies)		8 (14.54%)	1 (1.92%)	0.032
Shock Index at admission	0.7-0.9	28 (50.90%)	32 (61.53 %)	0.06
	1.0-2.0	26 (47.27%)	15 (28.84%)	
	>2	1 (1.81%)	5 (9.61%)	

Atonicity of the uterus was the most common cause of PPH, followed by genital tract trauma, retained products of conception, and coagulation disorders. Both medical and surgical means of management were used in our patients. Twenty-eight PRE patients (65.4%) and 34 POST patients (61.5%) required only medical management. Twenty-seven (34.6%) PRE patients and 18 POST patients (38.5%) required medical and surgical intervention. No patients received surgical intervention alone without medical intervention (χ2=2.29; p=0.129).

The article "Implementation of Postpartum Hemorrhage Emergency Care Using a Bundle Approach at a Tertiary Care Hospital in North India" was retracted in 2022. Reasons: errors in the text; concerns about the authorship.

Thirty-nine patients (75%) in the POST group received the first response bundle treatment (i.e., with intravenous [IV] fluids, uterine massage, TXA, and oxytocics), and 13 patients (25%) received the refractory bundle response. There was no significant increase in additional doses of uterotonics apart from standard doses of 20 units of IV oxytocin (p=1). There is a significant more than two-fold increase in the use of TXA in the POST group (32.69% vs. 12.72% in the PRE group) after the implementation of bundles (p=0.041).

Fifty-four patients (98.2%) required blood component transfusion in the PRE group, while 20 patients in the POST group (38.5%) required transfusion. Among PRE patients, 22 (40%) required only packed red blood cells (PRBC), five (9.1%) required only fresh frozen plasma (FFP), and 27 (49.1%) required both PRBC and FFP. Among POST patients, 15 (28.9%) required packed RBC, but the total consumption of blood components significantly declined by 60% in the POST group (p=0.0319). The requirement for radical surgical treatment of PPH, which included hysterectomies, was also significantly reduced, from 27.27% in the PRE group to 11.54% in the POST group (p=0.032).

Among PRE patients, 28 (50.9%) had an SI in the range of 0.7 to 0.9, 26 patients (47.3%) were in the range of 1.0 to 2.0, and one patient had an SI >2. For POST patients, 32 (61.5%) had an SI from 0.7 to 0.9, 15 patients (28.8%) had an SI of 1.0 to 2.0, and five (9.6%) had an SI >2 (χ2=5.81; p=0.06).

In the PRE period, the maternal mortality in the PPH patients was 3.3% (two out 61; 95% CI=0.9% to 11.2%), while in the POST period it was 1.75% (one out 57; 95% CI=0.31% to 9.3%), a NNT=64.5. There was no significant difference found (χ2=0.002; p=0.96). The odds of PPH non-occurrence after pre- and post-test was 1.103 (95% CI=0.747 to 1.635).

## Discussion

Care bundles have been employed to give high-quality clinical care by ensuring adherence to selected guidelines and procedural improvements. The "initial response to PPH bundle" and the "response to refractory PPH bundle" were developed by the WHO in 2017 as two care bundles of clinical therapies for PPH [10]. Uterotonics, IV fluids, TXA, and uterine massage were all part of the first PPH reaction bundle and were meant to be presented alongside supportive features including advocacy, training, teamwork, communication, respectful treatment, and the implementation of best clinical practices, like any other clinical bundle [10,13].

The article "Implementation of Postpartum Hemorrhage Emergency Care Using a Bundle Approach at a Tertiary Care Hospital in North India" was retracted in 2022. Reasons: errors in the text; concerns about the authorship.

The most important study assessing the success of an obstetric hemorrhage bundle was conducted in the California Maternal Quality Care Collaborative. A comprehensive maternal hemorrhage protocol was initiated within a health care system with 29 different delivery units and more than 60,000 annual births. Those hospitals varied in size, from small rural centers with 200 deliveries per year to large urban hospitals with >6,000 births annually. Their primary outcomes were the total number of units of blood transfused and the number of peripartum hysterectomies, which from baseline to 10 months post-implementation was reduced from 35.9 per 1,000 deliveries to 26.6 overall [14].

There is little evidence regarding the challenges of implementing care bundles in low- and middle-income countries. Therefore, we conducted a comparative study of PPH in patients before and after implementing the bundle care approach in our institute. We diagnosed more cases as mild or severe PPH after training. However, it is possible that our institute had one case of moderate PPH in that period or that mild and moderate cases of PPH were referred to our facility.

After the PPH care bundle implementation, we saw a significant decrease in the number of patients requiring blood components, and the consumption of blood products dropped significantly by 60% (p=0.0319). Reducing the demand for blood is critical in low-income countries, where the availability and use of blood product resources substantially influence PPH mortality. Some patients are transfused primarily for symptom alleviation because they have significant baseline anemia. We also reported that the number of women who needed radical surgery to treat PPH, such as hysterectomies, was significantly reduced by more than two times, from 27.27% in the PRE group to 11.5% in the POST group (p=0.032). Blood transfusion and radical surgeries are frequently employed as a marker for maternal morbidity associated with PPH.

To implement the bundle care approach, behavioral motivation and educational support are required among health care workers. The implementation requires clinical interaction at a multidisciplinary level [13,15,16]. The supporting elements are essential to the bundle's success. New guidelines for care bundles are unlikely to result in enhanced treatment quality [15,16]. However, sustainable guidelines, positive, supportive leadership, resource availability and proper use, training of medical personnel, teamwork, communication, record keeping, and focus on the quality of care are all factors that support or enable bundle implementation. Hospitals struggle to implement these recommendations due to time and resource constraints, multidisciplinary teamwork, and cultural shifts in working [17,18].

The article "Implementation of Postpartum Hemorrhage Emergency Care Using a Bundle Approach at a Tertiary Care Hospital in North India" was retracted in 2022. Reasons: errors in the text; concerns about the authorship.

Strengths and limitations

This study tries to address to a certain extent the paucity of research on the outcomes, the benefits and the difficulties involved in the successful execution of the bundle care approach in the management of PPH, more so in resource-limited situations. However, some important limitations of this study include confounding factors like age and parity not being accounted for and the comparison groups not being demographically equivalent, thereby accounting for the limited external validity of the results. Additionally, we noted observations immediately after TOT sessions that may affect bundle compliance. Hydration level affects hemoglobin level, which was used to calculate blood loss. Also, resource availability after training affects compliance with the implementation of the bundle care approach.

## Conclusions

This study was conducted to analyze whether implementing a PPH bundle of care may reduce maternal morbidity and mortality in our institution. The ideal goal of bleeding bundle establishment would be to lower the total rates of PPH and/or the total volume of blood lost per individual in PPH. While we noted a change in PPH management after bundle care training, the differences in outcomes were not always significant due to confounding factors. PPH care bundles retain the potential to improve the morbidity of PPH with fewer resources used and fewer interventions required. Further studies are needed with a larger group of patients that eliminate confounding factors to determine if PPH care bundles have comparable effects.
